The article "Computational Intelligence Powered Performance Analysis on Phase Change Heat Storage Air Source Heat Pump System" was published in 2022. Journal: Comput Intell Neurosci.

# Computational Intelligence Powered Performance Analysis on Phase Change Heat Storage Air Source Heat Pump System

**DOI:** 10.1155/2022/8906838

**Published:** 2022-08-04

**Authors:** Caihong Yin, Ronghua Wu, Hao Zhan, Hao Yu, Changqing Liu

**Affiliations:** ^1^Jiaozhou Bureau of Science, Technology and Industrial Information, Qingdao, Shandong 266399, China; ^2^Qingdao Kechuang Blue New Energy Co., Ltd, Qingdao, Shandong 266300, China; ^3^College of Mechanical and Electrical Engineering, Qingdao University, Qingdao, Shandong 266071, China

## Abstract

Aiming at the performance deterioration of air source heat pump at low temperature in cold area, an air source heat pump system with sodium chloride aqueous solution as low temperature phase change heat storage material was proposed to increase the air inlet temperature of the unit under low temperature conditions and improve the low temperature performance of the heat pump unit. The system form, unit energy consumption model, and economic model were given, and the operating economy of the traditional electric auxiliary heat air source heat pump system and the phase change heat storage air source heat pump system were compared through computational intelligence powered methods. On this basis, the operation economy of the heat pump system using different concentrations of sodium chloride solution as the heat storage material was simulated and optimized, and the operation efficiency and energy-saving performance of the system were analyzed by taking an actual residential building in a cold area as an example. The simulation results showed that the Heating Seasonal Performance Factor (HSPF) of the heat pump system using 8.5% sodium chloride aqueous solution as the heat storage material is 2.24, and the HSPF of the traditional electric auxiliary heat pump system is 1.83. Compared with the traditional electric auxiliary heat pump system, the phase change heat storage heat pump system saves heating energy consumption by 19.6% and defrosting energy consumption by 38.8%. The heat pump system using 10% sodium chloride aqueous solution as the heat storage material has the best operating economy, and the system HSPF is 2.33, which saves heating energy consumption by 23.2% and defrosting energy consumption by 34% compared with the traditional heat pump system. The operation condition of phase change heat storage air source heat pump system is stable, and the system performance is significantly improved.

## 1. Introduction

Air source heat pump is widely used in building heating and domestic hot water supply from renewable air. Heat pump takes heat from low temperature heat source based on the inverse Carnot cycle, and its condensation temperature is related to building heating requirements. In recent years, the promotion of energy-saving buildings reduces the heat standard for heating, but in order to ensure better heating comfort and heat transfer efficiency, the water supply temperature of radiant floor heating is still recommended to remain above 40°C [1]. The evaporation temperature of the heat pump changes with the outdoor temperature and maintains a certain degree of superheat. When the evaporation temperature decreases due to the decrease of the outdoor temperature, the compressor needs to consume more electrical energy to improve the compression ratio to keep the condensation temperature constant, and both the heating capacity and COP of the heat pump will be significantly attenuated at lower ambient temperature [2].

The article "Computational Intelligence Powered Performance Analysis on Phase Change Heat Storage Air Source Heat Pump System" was published in 2022. Journal: Comput Intell Neurosci.

Scholars in various countries have done a lot of research on improving the low temperature performance of air source heat pump and put forward a variety of solutions, which mainly focus on the structural improvement of the heat pump itself and the coupling of multiple heat sources in two aspects. The structural improvement of air source heat pump system operating in cold regions includes exploring new technologies and applying new working medium. Ji et al. [3] conducted an experimental study on the heating performance of a two-stage variable speed scroll compressor jet assisted air source heat pump, and the results showed that when the ambient temperature was reduced to −20°C, the system was still able to achieve 68.1% of the nominal working condition, and it could operate stably in severe cold regions. Lx et al. [4] experimentally verified the operational stability of the cascade air source heat pump system when it was applied in cold regions, and the results showed that the system operated stably in the heating season, and the efficiency was much higher than that of the gas boiler. Wu et al. [5] proposed and theoretically validated a new H_2_O/ionic liquid absorption and CO_2_ compressed air source heat pump system for ultra-low ambient temperature, which operated well at −30°C ambient temperature, and the primary energy efficiency (PEE) was higher than 1.256. Zhang et al. [6] simulated the heating performance of the cascade air source heat pump system using R134a/CO_2_ in severe cold regions. The simulation results showed that the HSPF of the system in the heating season remained above 2.1, and the system had high economy and reliability.

Compared with the traditional air source heat pump heating system, the design and control technology of the heat pump unit with two-stage compressor and cascade system are still not mature [7], and the operating efficiency at room temperature is far lower than that of the conventional heat pump unit. The promotion of new low-temperature working materials such as CO_2_ is limited due to the low unit heat load and high requirements for pressure vessels. At present, engineering applications more often use multiple heat sources coupled heating methods to reduce the operating time of heat pump units under unfavorable operating conditions. Sager and Poirier [8] conducted a field evaluation of the performance and cost competitiveness of a dual-source solar-assisted air source heat pump in cold climate, and the results showed that the system operated stably in cold climate, effectively reduced carbon emissions, and shortened the payback period. Sun et al. [9] combined electric boiler with air source heat pump to reduce the heating load of air source units in severe cold climate by peak shaving of electric boiler. The actual heating area of the system was 130650 m^2^, and the heating equipment operated stably. Zhao et al. [10] designed a gas-air dual-source heat pump to replace the existing gas boiler. When the ambient temperature decreases, and the electrical price ratio of the equivalent heating capacity is lower than 0.45, the unit takes heat from natural gas, which can effectively reduce the energy consumption of heating. In addition, there are also projects that deploy air source heat pump and water source heat pump at the same time to adjust the unit load ratio according to the outdoor temperature, with good energy saving effect [11].

The article "Computational Intelligence Powered Performance Analysis on Phase Change Heat Storage Air Source Heat Pump System" was published in 2022. Journal: Comput Intell Neurosci.

Heat storage technology can realize the transfer of heat in time and space. Adding heat storage system to air source heat pump system can further shorten the operation time of the heat pump under unfavorable working conditions and improve the low temperature performance of the unit. Chen et al. [12] conducted an experimental study on solar-air source heat pump system with heat storage device, and the results showed that the utilization of solar heat storage for heating at cold night could reduce the heating demand for the unit and effectively reduce the energy consumption of the unit. The COP of the system in extreme weather was maintained above 1.7. Different from most studies that directly applied solar energy heat to heat storage, Zhang et al. [13] used solar energy to preheat the cold air entering the evaporator. By increasing the dry-bulb temperature of the air and reducing the moisture content of the air, the evaporation temperature of the unit was increased, and the frosting was delayed. The system also paralleled the electric heating device behind the solar collector to preheat the air at night when the ambient temperature was low. The results showed that the system reduced the operation cost by 66.3%, resulting in significant energy saving effect. On the basis of the above system, Xu et al. [14] eliminated the electric heating device and replaced it with a heat storage tank after the condenser of the system. The unit operated at full load in the daytime and stored the surplus heat through the tank for nighttime heating, so that the unit did not operate or operated less at night, reducing the energy consumption of the unit, and reducing the number of units and unit investment.

The article "Computational Intelligence Powered Performance Analysis on Phase Change Heat Storage Air Source Heat Pump System" was published in 2022. Journal: Comput Intell Neurosci.

Common heat storage technologies include sensible heat storage, latent heat storage, and electrochemical heat storage, among which latent heat storage has high heat storage density, small footprint, and stable chemical properties, which has become a hot research topic in recent years [15]. The heat storage technology based on heat pump system includes condensation side heat storage and evaporation side heat storage. The most commonly used condensation side heat storage material is paraffin [16], which is chemically stable and relatively inexpensive, with stable crystallization and no supercooling problem compared with hydrated salt [17]. The heat storage temperature of the evaporation side is generally below 0°C, which is lower than the freezing point temperature of water. Therefore, most of the ice with low cost and high heat storage density is used as the heat storage material. The melting point temperature of the solution can be flexibly changed by adding inorganic salts or organic solutes to the water. Since the freezing of salt solution has the characteristics of water molecules precipitation and then solidification, the heat storage density of fluidized ice formed by mechanical stirring and other measures is high, and the heat transfer coefficient is much higher than that of ordinary solid ice. Sidqy et al. [18] proposed a process for making ice slurry from saline seawater by scraper method. Lee and Kim [19] produced an ice slurry heat storage device with mass density of 25% by adding 6.5% ethylene glycol solution into water. Sasaki [20] applied this property to the heat storage of distribution refrigerator and achieved good results.

Adding new heat sources to the existing air source heat pump heating projects is not easy to achieve, and most regions do not have the conditions of applying water source heat pump and industrial waste heat. Adding electric boilers and gas boilers is not in line with the concept of energy saving and environmental protection, so it is difficult to get government approval. Solar air preheating can effectively reduce the operation time of the unit under adverse conditions, but large-scale utilization of solar energy needs to lay a large area of collectors, and most old projects do not have implementation conditions. Therefore, based on not changing the old conventional air source heat pump module as much as possible, this paper proposes an air source heat pump system that uses the fluidized ice heat storage technology to store end heat for preheating cold air entering the evaporator in extremely cold weather. The heat is stored when the thermal efficiency of the unit is high in rising temperatures and released when the thermal efficiency of the unit decreases in extremely cold weather, ensuring that the unit always maintains a low compression ratio, reducing the heating energy consumption and, at the same time, reducing the investment in peak heat spare units. The system form, unit energy consumption model, and the economic model were given in the paper. The operating characteristics of the traditional air source heat pump system and the new heat pump system were compared by means of numerical analysis. On this basis, the operating economy of the heat pump system with different heat storage temperatures was simulated and optimized. Taking a residential building heating project in Dalian as an example, the system performance of the traditional heat pump heating and the new heat pump heating was compared by means of numerical analysis, and the optimal operating point of the system running in the residential area was found.

The article "Computational Intelligence Powered Performance Analysis on Phase Change Heat Storage Air Source Heat Pump System" was published in 2022. Journal: Comput Intell Neurosci.

## 2. Introduction of Phase Change Heat Storage Air Source Heat Pump System

Since the design of the existing air source heat pump unit has been extremely mature, in order to adapt widely to the existing air source heat pump units, the phase change preheating system preheats the air by extending the air duct and then adding part of finned heat exchanger tubes at the bottom of evaporator without changing the existing structure of heat pump units and influencing the fluorine circuit cycle. When the air temperature is high, and the operating efficiency of the unit is high, such as during the day, the intermediary water is used to take heat from the end to melt the ice crystals in the heat storage device, so as to achieve the purpose of heat storage. When the outdoor temperature is low, and the unit efficiency is reduced, for example, at night, the intermediate water takes heat from the heat storage device to preheat the evaporator intake to improve the low-temperature performance of the unit. The schematic diagram of the system is shown in Figure 1.

When the outdoor temperature is low, and the operating efficiency of the air source heat pump unit decreases, open solenoid valve 1 and solenoid valve 3, and close solenoid valve 2. The intermediate antifreeze takes heat from the heat storage device through the intermediate pump and uses the finned heat exchanger tube to heat the intake air, improves the operating conditions of the unit under low ambient temperature, and increases the heating capacity of the unit.

The article "Computational Intelligence Powered Performance Analysis on Phase Change Heat Storage Air Source Heat Pump System" was published in 2022. Journal: Comput Intell Neurosci.

When the outdoor temperature warms up, and the energy efficiency of the unit is high, close solenoid valve 3, open solenoid valve 1 and solenoid valve 2, and heat is taken from the intermediate water at end by the end pump, which is used for ice melting and heat storage.

Electric auxiliary heating air source heat pump system uses electric boiler as auxiliary heat source and provides heat by parallel connection of conventional air source heat pump unit and electric boiler. The outdoor design temperature of air source heat pump unit is −10°C. Start the electric boiler when the outdoor ambient temperature is lower than −10°C. It serves as the supplementary heat source after attenuation of heat generation of heat pump system under low temperature conditions.

Figure 2 is the typical air enthalpy and humidity diagram of the two heating methods. The curve ABC represents the change of air enthalpy and humidity on the surface of the evaporator fins of the conventional heat pump unit. During the process from A to B, the sensible heat of outdoor air releases heat, and the moisture content increases, while the temperature decreases. When the outdoor air reaches the state point B, it reaches the saturated humidity. From B to C, the air temperature gradually decreases, and the water vapor in the air continuously precipitates and condenses, condensing and frosting on the surface of the evaporator [21]. There are both sensible and latent heat release in this process.

The curve DEF represents the change of air enthalpy and humidity on the surface of evaporator fins of the regenerative air source heat pump unit when the heat accumulator releases heat. During the process from D to E, the air flows through the preheating fins to absorb heat, and the temperature rises. Because there is no mass transfer process in the wall-type heat exchange, the moisture content of the air will not change, and the actual moisture content of the air will decrease. During the process from E to F, the air flows through the fluorine path fins, the temperature decreases, and the moisture content increases, but it does not reach the saturated moisture content of point F. There is only sensible heat exchange in the entire heat exchange process, and there is no risk of frosting.

## 3. Energy Consumption Model of Air Source Heat Pump

In order to further analyze the low temperature performance of the phase change heat storage heat pump system, an energy consumption model of air source heat pump was established [22]. In the heating season, the outdoor performance balance point temperature of −10°C is selected as the design temperature [23], and the condensation temperature of the unit is 50. The operating range of a certain brand of scroll heat pump unit using R410A as the working medium is shown in Figure 3. The compressor rated suction and discharge capacity is 0.394 kg/s. According to the operating range provided by the manufacturer, the conventional heat pump unit cannot work normally when the evaporation temperature is lower than −15°C.

The article "Computational Intelligence Powered Performance Analysis on Phase Change Heat Storage Air Source Heat Pump System" was published in 2022. Journal: Comput Intell Neurosci.

As a pressure regulating component, the state change of the refrigerant in the compressor is a transient process, Therefore, it is assumed that (1) the state of the refrigerant in the compressor is independent of the time constant [24], and its change process can be ignored compared with that in the heat exchanger; (2) the compression process of the refrigerant in compressor is isentropic [25]. Therefore, the steady-state characteristics of the unit can be used instead of dynamic characteristics. The performance parameters such as the power consumption and heating capacity of the compressor are affected by evaporating temperature and condensing temperature. According to the actual operating parameters of the compressor, the Coefficient of Performance (COPcomp) curve of its operating energy efficiency can be obtained as follows:

(1) $$\begin{array}{c} {\text{COP}}_{\text{comp}}=7.3562+0.09181\left(t_{\text{air}}-t_{\text{sh}}\right)-0.09716\left(t_{\text{c}}+t_{\text{sc}}\right), \end{array}$$

where *t*_air_ is the intake air temperature, °C; *t*_sh_ is the degree of superheat, °C; *t*_*c*_ is the unit outlet water temperature, °C; *t*_*sc*_ is the degree of supercooling, °C.

According to the product sample book, the rated water flow of the selected air-cooled heating module is 22.4 m^3^/h, the total air volume of the fan is 48000 m^3^/h, and the pump power *P*_aspw_ and the fan power *P*_aspa_ are

(2) $$\begin{array}{c} P_{\text{aspw}}=\frac{G_{w}g\rho H}{3600\eta_{\text{pw}}},\\ P_{\text{aspa}}=\frac{Q_{\text{air,in}}P_{\text{air}}}{3600\eta_{\text{pa}}}, \end{array}$$

where *G*_*w*_ is the water flow rate of unit, m^3^/h; *g* is the acceleration of gravity, 9.8 m/s^2^; *ρ* is the fluid density, kg/m^3^; *H* is the head, *m*; *η*_pw_ is the pump efficiency, 0.85; *Q*_air,in_ is the intake air volume, m^3^/h; *P*_air_ is the total pressure, kPa; *η*_pa_ is the full pressure efficiency, 0.85.

The unit adopts the hot gas bypass method of four-way valve reversing for defrosting [26]. According to the research results of Qu et al. [27], the energy consumption of melting and defrosting accounts for about 15.7% of the energy consumption of defrosting [27], and the evaporation of water for melting and defrosting is about 13% [28]. The defrosting energy consumption of the unit *P*_def_ is

(3) $$\begin{array}{c} P_{\text{def}}=\frac{Q_{\text{air}}\left(d_{\text{air,in}}-d_{\text{air,out}}\right)}{565200}\gamma , \end{array}$$

where *d*_air,in_ is the average moisture content of the intake air, g/m^3^; *d*_air,out_ is the average moisture content of the exhaust gas, g/m^3^; *γ* is the coagulation heat of water, kJ/kg.

The article "Computational Intelligence Powered Performance Analysis on Phase Change Heat Storage Air Source Heat Pump System" was published in 2022. Journal: Comput Intell Neurosci.

Under low temperature conditions, the heating capacity of the heat pump unit is used to meet the building heat load demand. After the ambient temperature is increased, part of the heating capacity of the heat pump unit is used for ice melting and heat storage of the heat storage device. The actual heating energy consumption *P*_asp_ of the unit is

(4) Pasp=Paspw+P+aspaPdef+qload/ηasp+qPCM/ηPCMCOPcomp,

where *q*_load_ is the building heat load corresponding to ambient temperature, kW; *q*_PCM_ is the heat storage load, kW; *η*_asp_ is the unit heat transfer efficiency, 0.95; *η*_PCM_ is the heat storage heat transfer efficiency, 0.9.

## 4. Energy Consumption Model of Phase Change Heat Storage Device

The phase change heat storage device adopts the ice crystal cold storage technology of dynamic crystallization [29, 30], and the heat exchange area on both sides is 20 m^2^. Dynamic crystallization overcomes the problems of high supercooling degree, wall thermal resistance increasing with the amount of ice and ice blockage of pipeline existing in traditional static ice storage technology. The phase change heat storage material is a certain concentration of sodium chloride salt solution, and a mechanical stirring structure is set inside the device to ensure that the subcooling degree of the salt solution is consistent, so that the freezing process occurs homogeneously. Adjusting the mass concentration of sodium chloride in the solution can change the temperature of the phase transition point of the device (supercooled crystallization temperature of sodium chloride solution), and the approximate formula [31] of the crystallization point temperature T_crys_ of sodium chloride aqueous solution is

(5) $$\begin{array}{c} T_{\text{crys}}=-36.97w^{2}-57.28w+0.1037, \end{array}$$

where *w* is the mass concentration of sodium chloride, %.

The partially crystallized sodium chloride solution is in a two-phase flow state in the device and has high fluidity [32]. Compared with the traditional static ice storage technology, the ice crystal cold storage can realize the continuous crystallization of the cold storage device, and the ice crystal in the solution has a higher specific surface area for heat exchange. The heat transfer coefficient of ice slurry with ice content of 5w%∼30w% is about 3 kW/(m^2^·K), and the heat of solution is about 334 kJ/kg. In order to simplify the calculation process, the following assumptions are made for the phase change heat storage process: (1) the pressure drop and heat loss of intermediary water in the regenerator are ignored in the modeling process; (2) intermediate water flows in all directions in the heat accumulator; (3) the equivalent specific heat capacity method is used to describe the phase transition process of phase change materials [25]. Based on the above assumptions, the heat transfer process of the phase change side of the accumulator is as follows:

(6) $$\begin{array}{c} \left\{\begin{array}{c} E_{\text{PCMch,sc}}\int_{0}^{\tau_{ch}}k_{\text{PCM,sc}}A_{\text{PCM,sc}}\left(t_{\text{ave,sc}}-t_{\text{PCM,sc}}\right)\text{d}\tau ,\\ E_{\text{PCMch,pc}}\int_{0}^{\tau_{ch}}k_{\text{PCM,pc}}A_{\text{PCM,pc}}\left(t_{\text{ave,pc}}-t_{\text{PCM,pc}}\right)\text{d}\tau ,\\ E_{\text{PCMch,cc}}\int_{0}^{\tau_{ch}}k_{\text{PCM,cc}}A_{\text{PCM,cc}}\left(t_{\text{ave,cc}}-t_{\text{PCM,cc}}\right)\text{d}\tau , \end{array}\right. \end{array}$$

where *E*_PCMch_ is the heat storage of phase change material, kJ; *k*_PCM_ is the heat transfer coefficient of phase change side, W/(m^2^·K), calculated according to Dittus-Boelter formula; *A*_PCMch_ is the heat transfer area on phase change side, m^2^; *t*_ave_ is the average temperature of tube wall, °C; *t*_PCM_ is the average temperature of phase transition side, °C; *τ*_ch_ is the heat storage time, *h*; subscript: sc is the overheating stage; pc is the two-phase stage; cc is the supercooling stage.

The article "Computational Intelligence Powered Performance Analysis on Phase Change Heat Storage Air Source Heat Pump System" was published in 2022. Journal: Comput Intell Neurosci.

Intermediate side heat transfer process:

(7) $$\begin{array}{c} E_{\text{tr},\text{in}}=m_{\text{tr}}\left(h_{\text{tr},\text{out}}-h_{\text{tr},\text{in}}\right)=k_{\text{tr}}A_{\text{tr}}\left(t_{\text{tr},\text{out}}-t_{\text{tr},\text{in}}\right), \end{array}$$

where *E*_tr,in_ is the heat storage capacity, kW; *m*_tr_ is the intermediate water flow, kg/s; *h*_tr,out_ is the outlet enthalpy, kJ/kg; *h*_tr,in_ is the inlet enthalpy, kJ/kg; *k*_tr_ is the heat transfer coefficient of intermediate water side, kW/(m^2^·K); *A*_tr_ is the heat exchange area of intermediate water side, m^2^; *t*_tr,out_ is the outlet water temperature, °C; *t*_tr,in_ is the inlet water temperature, °C.

The energy consumption of phase change heat storage device is

(8) $$\begin{array}{c} P_{\text{PCM}}=P_{\text{PCM},\text{motor}}+q_{\text{PCM}}\left(1-\eta_{\text{PCM}}\right), \end{array}$$

where *P*_PCM,motor_ is the motor power, kW.

The finned tube side adopts traditional dry air-cooled finned heat exchanger, and the heat exchange *E*_fin,evap_ is

(9) $$\begin{array}{c} E_{\text{fin,evap}}=m_{\text{fin}}\left(h_{\text{fin,in}}-h_{\text{finout}}\right)=k_{\text{fin}}A_{\text{evap}}\left(t_{\text{fin,in}}-t_{\text{fin,out}}\right), \end{array}$$

where *M*_fin_ is the water flow in the pipe, kg/s; *h*_fin,in_ is the inlet enthalpy, kJ/kg; *h*_fin,out_ is the outlet enthalpy, kJ/kg; *k*_fin_ is the fin heat transfer coefficient, W/m^2^; *A*_evap_ is the fin heat exchange area, m^2^; *t*_fin,in_ is the intermediate inlet water temperature, °C; *t*_fin,out_ is the intermediate outlet water temperature, °C.

Air side temperature change *δt* is

(10) $$\begin{array}{c} \delta t=\frac{3600E_{\text{fin,evap}}\rho_{\text{air}}}{Q_{\text{air,in}}c_{\text{air}}}, \end{array}$$

where *ρ*_air_ is the air density, kg/m^3^; *C*_air_ is the air specific heat capacity, kJ/(kg·K).

## 5. System Operation Energy Consumption Model

Heating Seasonal Performance Factor (HSPF) [33] is the ratio of the heating capacity and the total power consumption of the heat pump unit in a specific area during the normal heating season. At the same time, considering the steady-state efficiency, environmental changes, and the power consumption of the equipment other than the compressor of the unit, the HSPFasp calculation formula of the heat storage heat pump unit is

(11) $$\begin{array}{c} {\text{HSPF}}_{\text{asp,PCM}}=\frac{\int_{0}^{\tau_{\text{heat}}}q_{\text{load}}\text{d}\tau }{\int_{0}^{\tau_{\text{unit}}}P_{\text{asp}}\text{d}\tau }. \end{array}$$

The HSPF_auxi_ calculation formula of the electric boiler combined heating unit is

(12) $$\begin{array}{c} {\text{HSPF}}_{\text{auxi}}=\frac{\int_{0}^{\tau_{\text{heat}}}q_{\text{load}}\text{d}\tau }{\int_{0}^{\tau_{\text{unit}}}P_{\text{asp}}\text{d}\tau +\int_{0}^{\tau_{\text{boiler}}}P_{\text{boiler}}\text{d}\tau }, \end{array}$$

where *τ*_heat_ is the heating time in heating season, *h*; *τ*_unit_ is the heating time of heat pump unit, *h*; *P*_boiler_ is the power of auxiliary electric boiler, kW; *τ*_boiler_ is the heating time of auxiliary electric boiler, *h*.

Due to the long-term operation in the sub-zero environment, the saturated air moisture content decreases significantly with the decrease of temperature, and frequent defrosting is required during the operation of the unit. However, frequent defrosting not only affects the heating effect of the unit, but also greatly affects the operating energy efficiency of the unit. The influence of defrosting on the actual heating effect of the unit is mainly reflected in the proportion of defrosting time *x*_1_ and defrosting energy consumption *x*_2_:

(13) $$\begin{array}{c} x_{1}=\frac{\tau_{\text{def}}}{\tau_{\text{heat}}},\\ x_{2}=\frac{\int_{0}^{\tau_{\text{def}}}P_{\text{def}}\text{d}\tau }{\int_{0}^{\tau_{\text{heat}}}q_{\text{load}}\text{d}\tau }. \end{array}$$

The operation energy consumption of the electric boiler auxiliary air source heat pump system and the regenerative air source heat pump system is analyzed, mainly by comparing the primary energy consumption under the same outdoor working conditions and building load, and the low calorific value of standard coal(LHV_sc_ = 29.307 MJ/kg) [34] is introduced for this purpose, and the primary energy consumption PEC_EASP_ and utilization rate PER_EASP_ of the electric boiler auxiliary heating system are

(14) $$\begin{array}{c} \left\{\begin{array}{c} {\text{PEC}}_{\text{EASP}}=\frac{3600}{\eta_{E}}\times \left(\frac{\int_{0}^{\tau_{\text{unit}}}P_{\text{asp}}\text{d}\tau }{\eta_{\text{asp}}\cdot {\text{LHV}}_{\text{sc}}}+\frac{\int_{0}^{\tau_{\text{boiler}}}P_{\text{boiler}}\text{d}\tau }{\eta_{\text{boiler}}\cdot {\text{LHV}}_{\text{sc}}}\right),\\ {\text{PER}}_{\text{EASP}}=\eta_{E}\cdot \eta_{\text{asp}}\cdot \eta_{\text{boiler}}. \end{array}\right. \end{array}$$

PEC_PASP_ and utilization rate PER_PASP_ of the thermal storage air source heat pump system are

(15) $$\begin{array}{c} \left\{\begin{array}{c} {\text{PEC}}_{\text{PASP}}=\frac{3600\times \int_{0}^{\tau_{\text{unit}}}P_{\text{asp}}\text{d}\tau }{{\text{LHV}}_{\text{sc}}\cdot \eta_{\text{asp}}\cdot \eta_{E}},\\ {\text{PER}}_{\text{PASP}}=\eta_{\text{asp}}\cdot \eta_{\text{PCM}}\cdot \eta_{E}, \end{array}\right. \end{array}$$

where *η*_*E*_ is the thermoelectric efficiency, 0.42.

The article "Computational Intelligence Powered Performance Analysis on Phase Change Heat Storage Air Source Heat Pump System" was published in 2022. Journal: Comput Intell Neurosci.

## 6. Performance Comparison and Optimization of Heat Storage Heat Pump System and Electric Auxiliary Heat Pump System

A residential building with a heating area of 3000 m^2^ in Dalian is selected as the main heating body. The building envelope, fresh air demand internal personnel, lighting, and other thermal disturbance factors are in accordance with the provisions of GB50189 “Energy-saving Design Standards for Public Buildings.” The specific design parameters are shown in Table 1.

When the indoor temperature is maintained at 18°C, and the outdoor environment temperature changes from −15°C to 14°C, the scatter diagram of the change of building heat load with outdoor ambient temperature is obtained by using transient analysis software, as shown in Figure 4.

It can be seen from Figure 4 that the actual heat load of the building has an almost linear relationship with the outdoor temperature. When the outdoor temperature is 14°C, the building heat load is only 18 kW. With the decrease of outdoor temperature, the heat dissipation of the building gradually increases. When the outdoor temperature drops to −14°C, the maximum heat load of the building reaches 157 kW, at which time the heat demand of the building is the largest, and the heating capacity of the unit is the smallest. From the density of the scatter plot, it can be found that the concentration of building heat load is small in the area above 0°C. At this time, due to the small temperature difference between the inner and outer surfaces of the wall, the building heat dissipation is greatly affected by meteorological factors other than ambient temperature, such as solar radiation, rain, and snow. When the ambient temperature is lower than −10°C, the heat load distribution of the building is relatively concentrated. The heat loss of the building is mainly due to heat exchange with outdoor air in areas such as walls and windows. The influence of solar radiation on the heat dissipation of the building can be approximately ignored. The design of energy-saving buildings can also refer to this result and reduce the heating load of the building by installing double glazing and increasing the thickness of the insulation layer.

### 6.1. Performance Comparison between Heat Storage Heat Pump System and Electric Auxiliary Heat Pump System

Numerical simulation of the heating performance of the electric auxiliary heating air source heat pump system and the regenerative air source heat pump heating system is carried out in a typical meteorological year [26] in Dalian. Referring to the heating season time in Dalian, the simulation time was set from November 5 of the current year to April 5 of the next year, and in order to reduce the calculation amount and ensure the calculation accuracy, 1 h is taken as a time step. The simulation takes 1 h as a step. The sodium chloride solution with a mass concentration of 8.5% is selected as the phase change heat storage material. According to formula (6), the corresponding crystal phase transition point temperature of the sodium chloride solution of this concentration is −5°C. The change of HSPF of two heating methods with heating time in the heating season is shown in Figure 5:

It can be seen from the figure that the outdoor ambient temperature is high before the 1100 h of heating, that is, December 21, and the HSPF of the two heating methods is relatively close. After December 21, the outdoor ambient temperature decreases, and the heat storage heat pump system maintains the HSPF above 1.74 through heat storage and peak regulation. The average HSPF in the heating season is 2.24, while the minimum HSPF of the electric auxiliary heat pump system is 0.95, and the average heating HSPF in the heating season is 1.83. The HSPF of the electric auxiliary heat pump system is lower than 1 because the heating capacity of the unit is greatly attenuated under extremely cold conditions, and the electric boiler with lower thermal efficiency bears most of the night heat load.

The article "Computational Intelligence Powered Performance Analysis on Phase Change Heat Storage Air Source Heat Pump System" was published in 2022. Journal: Comput Intell Neurosci.

Comparing the variation law of defrosting energy consumption with heating time of the two heating methods under frosting conditions, the results are shown in Figure 6.

It can be seen from the figure that the defrosting energy consumption curves of the two heating methods have similar trends. In the period from 0 h to 1000 h, that is, from November 5 to December 17, the outdoor temperature hovered around 0°C, the outdoor air moisture content is large, the frosting on the surface of the fin is fast and the frosting amount is large [35], and the defrosting energy consumption increases rapidly. And due to the short operating time of the heat storage device at this temperature, the defrosting energy consumption of the heat storage heat pump system is not significantly reduced. With the continuous decline of outdoor temperature and the decrease of air moisture content, the increasing trend of defrosting energy consumption of both systems is slowing down [35]. Due to the long-term operation of the heat storage device in the heat storage pump system under low temperature environment, the moisture content of the air is further reduced, and the frosting amount at the same time is reduced. In fact, the defrosting energy consumption of the system is less, and the difference between the defrosting energy consumption of the two systems is gradually enlarged. According to the simulation results, in the whole heating season, the defrosting energy consumption of the heat storage heat pump system is 1287 kW·h, and the total defrosting time is 330 h, accounting for 9.3% of the unit operating time. Compared with the electric auxiliary heat pump system, the defrosting energy consumption is reduced by 816 kW·h, and the defrosting downtime is reduced by 131 h. The simulation results show that the primary energy consumption of the heat storage heat pump system in the whole heating season is 47822kgcc, which saves 19.6% of the primary energy compared with the traditional electric auxiliary heat pump system.

### 6.2. Performance Optimization of Phase Change Heat Storage Air Source Heat Pump System

In order to further optimize the performance of the heat storage air source heat pump system and analyze the actual energy consumption performance of the system, adjust the concentration of sodium chloride salt in the heat storage device appropriately. The temperature of the phase transition point of the heat storage device is changed with a step size of 1°C, and the change of HSPF and the primary energy consumption of the system under different temperatures are obtained as shown in Figure 7. The cumulative heat storage and defrosting energy consumption in the heating season are shown in Figure 8.

The article "Computational Intelligence Powered Performance Analysis on Phase Change Heat Storage Air Source Heat Pump System" was published in 2022. Journal: Comput Intell Neurosci.

According to Figure 7, the HSPF of the heat storage heat pump system shows a trend of first increasing and then decreasing with the decrease of the heat storage temperature, and the primary energy consumption is the opposite. Although the energy efficiency ratio of the heat pump unit increases with the increase of the intake air temperature after preheating, it can be seen from Figure 8 that, with the increase of the phase transition point temperature, the accumulated heat storage in the heating season also increases. Due to the mechanical loss in the heat storage process of the heat storage device, and the heat loss in the heat storage and heat release process, the increase of the HSPF of the unit with the increase of the phase transition point temperature has a certain limit. The heat loss from heat storage caused by the excessive high phase transition point temperature is greater than the electric energy saved by the improvement of the unit efficiency. When the phase transition point temperature is −5.9°C, the system has a maximum HSPF of 2.33, and the primary energy consumption is 45736kgcc, which is 23.2% less than the electric auxiliary heat pump system. The defrosting energy consumption of the unit decreases with the decrease of the phase transition point temperature, and the decreasing trend gradually slows down. The analysis is because the low temperature air has a low moisture content. When the air temperature is lower than −9°C, the amount of frost itself is very small, and the amount of frost that is reduced by thermal storage preheating does not account for a small proportion of the total amount of frost.

## 7. Conclusion

1. When the sodium chloride solution with a mass concentration of 8.5% is used as the phase change heat storage material, the average HSPF of the phase change heat storage air source heat pump system in the heating season is 2.24, which is 0.41 higher than that of the traditional electric auxiliary heat pump system. The primary energy consumption is 47852kgcc, the defrosting energy consumption is 1287 kW·h, which are 19.6% and 38.8% lower than those of the electric auxiliary heat pump system respectively, and the defrosting downtime is reduced by 28.4%.
2. When the sodium chloride solution with a mass concentration of 10% is used as the phase change heat storage material, the phase change heat storage heat pump system has the best system operation economy, and the average HSPF in the heating season of the system reaches 2.33, which reduces the defrosting energy consumption by 34% and saves primary energy by 23.2% compared with the traditional electric auxiliary heat pump system under the same working conditions.
3. The regenerative air source heat pump system using sodium chloride solution as the low-temperature phase change heat storage material operates stably, which can significantly reduce the energy consumption of defrosting and heating.
4. Due to the limitation of compressor capacity and noise problem, air source heat pump cannot be large-scale. When heating in large areas, dozens of units are generally used in parallel. When the number of parallel units is too large, or the spacing is too small, the mutual interference between suction and exhaust between units is likely to occur, resulting in obvious cold island effect [36]. At this time, even at a high outdoor temperature, the evaporation temperature of the unit in the middle position will also decrease sharply, resulting in the performance degradation of the unit. The numerical simulation in this paper relies on the mathematical model of a single unit, which cannot analyze the operating characteristics when multiple units are operated in parallel. Therefore, the existing mathematical model needs to be improved in the next step to increase the interference the interference component between different units for large-scale heating in order to investigate the energy saving performance of the system when applied to large-scale regional heating.

The article "Computational Intelligence Powered Performance Analysis on Phase Change Heat Storage Air Source Heat Pump System" was published in 2022. Journal: Comput Intell Neurosci.

## Figures and Tables

**Figure 1:** Operating principle diagram of phase change heat storage air source heat pump system. (1) Compressor. (2) Condenser. (3) Throttle valve. (4) Evaporator. (5) Four-way valve. (6) Fan. (7) End heat exchanger. (8) Phase change heat storage device. (9) End pump. (10) Intermediate pump. (11) Solenoid valve 1. (12) Solenoid valve 2. (13) Solenoid valve 3.

**Figure 2:** Air enthalpy and humidity diagram in the evaporator.

**Figure 3:** Compressor operating range.

**Figure 4:** Distribution of building heat load with ambient temperature.

**Figure 5:** The change of HSPF of two heating methods.

**Figure 6:** Comparison of defrosting energy consumption between two systems.

**Figure 7:** HSPF and primary energy consumption at different phase transition temperature.

**Figure 8:** Cumulative heat storage and defrosting energy consumption at different phase transition point temperatures.

**Table 1:** Building heat load design parameters.

Design parameter	
Heating system	Radiant floor heating
Supply and return water temperature/°C	45/35
Heat supply temperature/°C	18
Relative humidity/%	40
Building envelope	50% design standard for energy saving of public buildings
Number of occupants (person/m^2^)	0.18
Room rate of personnel	0.7

## Data Availability

The data used to support the findings of this study are available from the corresponding author upon request.
